RETRACTED

# Dclk1, a tumor stem cell marker, regulates pro-survival signaling and self-renewal of intestinal tumor cells

**DOI:** 10.1186/s12943-017-0594-y

**Published:** 2017-02-01

**Authors:** Parthasarathy Chandrakesan, Jiannan Yao, Dongfeng Qu, Randal May, Nathaniel Weygant, Yang Ge, Naushad Ali, Sripathi M. Sureban, Modhi Gude, Kenneth Vega, Eddie Bannerman-Menson, Lijun Xia, Michael Bronze, Guangyu An, Courtney W. Houchen

**Affiliations:** 1 Division of Digestive Diseases and Nutrition, Department of Medicine, University of Oklahoma Health Sciences Center, Oklahoma City, OK 73104 USA; 2 OU Cancer Institute, University of Oklahoma Health Sciences Center, Oklahoma City, OK USA; 3 Department of Veterans Affairs Medical Center, Oklahoma City, OK USA; 4 Access Endocrine, Diabetes and Thyroid center, Oklahoma City, OK USA; 5 Department of Medicine, National Jewish Health, Denver, CO USA; 6 Oklahoma Medical Research Foundation, Oklahoma City, OK USA; 7 Beijing Chao-Yang Hospital Department of Oncology, Capital Medical University, Beijing, China; 8 COARE Biotechnology, Oklahoma City, OK USA

**Keywords:** Dclk1, APC mutation, Cancer stem cells, Intestinal epithelial cells, Pro-survival signaling, Self-renewal, Nanoparticles, Colorectal cancer

## Abstract

**Background:**

More than 80% of intestinal neoplasia is associated with the *adenomatous polyposis coli* (*APC*) mutation. Doublecortin-like kinase 1 (Dclk1), a kinase protein, is overexpressed in colorectal cancer and specifically marks tumor stem cells (TSCs) that self-renew and increased the tumor progeny in *Apc* ^*Min/+*^ mice. However, the role of Dclk1 expression and its contribution to regulating pro-survival signaling for tumor progression in *Apc* mutant cancer is poorly understood.

**Methods:**

We analyzed DCLK1 and pro-survival signaling gene expression datasets of 329 specimens from TCGA Colon Adenocarcinoma Cancer Data. The network of DCLK1 and pro-survival signaling was analyzed utilizing the GeneMANIA database. We examined the expression levels of Dclk1 and other stem cell-associated markers, pro-survival signaling pathways, cell self-renewal in the isolated intestinal epithelial cells of *Apc* ^*Min/+*^mice with high-grade dysplasia and adenocarcinoma. To determine the functional role of Dclk1 for tumor progression, we knocked down Dclk1 and determined the pro-survival signaling pathways and stemness. We used siRNA technology to gene silence pro-survival signaling in colon cancer cells in vitro. We utilized FACS, IHC, western blot, RT-PCR, and clonogenic (self-renewal) assays.

**Results:**

We found a correlation between DCLK1 and pro-survival signaling expression. The expression of Dclk1 and stem cell-associated markers Lgr5, Bmi1, and Musashi1 were significantly higher in the intestinal epithelial cells of *Apc* ^*Min/+*^mice than in wild-type controls. Intestinal epithelial cells of *Apc* ^*Min/+*^mice showed increased expression of pro-survival signaling, pluripotency and self-renewal ability. Furthermore, the enteroids formed from the intestinal Dclk1^+^ cells of *Apc* ^*Min/+*^mice display higher pluripotency and pro-survival signaling. Dclk1 knockdown in *Apc* ^*Min/+*^ mice attenuates intestinal adenomas and adenocarcinoma, and decreases pro-survival signaling and self-renewal. Knocking down RELA and NOTCH1 pro-survival signaling and DCLK1 in HT29 and DLD1 colon cancer cells in vitro reduced the tumor cells’ ability to self-renew and survive.

RETRACTED

**Conclusion:**

Our results indicate that Dclk1 is essential in advancing intestinal tumorigenesis. Knocking down Dclk1 decreases tumor stemness and progression and is thus predicted to regulate pro-survival signaling and tumor cell pluripotency. This study provides a strong rationale to target Dclk1 as a treatment strategy for colorectal cancer.

**Electronic supplementary material:**

The online version of this article (doi:10.1186/s12943-017-0594-y) contains supplementary material, which is available to authorized users.

## Background

*APC* is a tumor suppressor gene that is mutated in patients with familial adenomatous polyposis (FAP) and most sporadic colorectal cancers [1, 2]. The *Apc* mutation dysregulates the Wnt signaling pathway and triggers cellular transformation, resulting in the development of adenomatous polyps [3]. It was suggested that the *APC* gene mutation is required, but is not sufficient, for the development of cancer in the colon. Since tumorigenesis is considered the result of multiple genetic changes, several efforts have made to identify those tumorigenesis-promoting changes. Several genetic changes, including activation mutations in *Ki-RAS/N-RAS*, mutations in the tumor suppressor *TP53*, and deletion of a region of chromosome 18 containing *SMAD2*, *SMAD4*, and *DCC* have been identified [4]. Despite improvements in our understanding of this disease, the molecular events underlying the development and progression of intestinal tumors are still largely unknown and may be a key to the development of more effective and novel therapeutic strategies. Therefore, understanding the *APC* gene mutation associated changes for intestinal tumorigenesis is important.

Similar to humans with germline mutations in *APC*, *Apc* ^*Min/+*^ mice have a heterozygous mutation in the *Apc* gene, predisposing the mice to intestinal and colon tumor development. These mice start developing intestinal polyps by ~4 weeks of age, with progression to dysplasia at 18–21 weeks; adenocarcinoma is also evident at ~26-34 weeks [5–8]. Eight-to-twelve-week-old *Apc* ^*Min/+*^ mice are a good model with which to study the pathogenesis of FAP, while 26-to-34-week-old *Apc* ^Min/+^ mice develop intestinal high-grade dysplasia and adenocarcinoma, and are a particularly relevant model for studying tumor progression and developing therapeutic strategies [6, 7]. *Apc* ^Min/+^ mice develop high-grade dysplasia and adenocarcinoma and are a clinically relevant disease model, since a large number of patients diagnosed with advanced colon cancer are elderly and have unresectable or widespread disease [9].

RETRACTED

Doublecortin-like kinase 1 (Dclk1) is a microtubule-associated protein kinase and has been identified as a tuft cell marker in the small intestine [10]. Dclk1 has been reported to mark tumor stem cells in the intestine and pancreas [11–15]. Emerging evidence has confirmed that the majority of human malignancies are initiated and maintained by a distinct population of cells that display stem cell properties and self-renewal ability [16]. More recently, it has been shown that the development and progression of colon and pancreatic cancer depend upon Dclk1^+^ cancer stem cells [11, 13–15]. We reported that Dclk1 is overexpressed in many cancers, including colon, pancreas, liver, and esophageal cancer [12, 17–20]. Previous work from others and us supported the idea that DCLK1 expression is critical for cancer stem cells, cancer growth, EMT, and metastasis [11, 12, 15, 18, 21–23]. These data provide a basis for Dclk1 as a regulatory factor for tumor growth and advancement.

Recent studies have indicated that neoplastic cells have active pro-survival signaling pathways for proliferation, resistance, self-renewal, and survival [24–26]. Furthermore, progression of cancer, including metastasis and secondary tumor formation of cancer cells with self-renewal ability, is often linked to altered expression of pro-survival signaling pathways [27]. Understanding the diversity of pro-survival signaling pathways that underlie cancer formation and progression is essential for developing a new generation of effective anticancer drugs for combinatorial therapeutic strategies. The interdependence between pro-survival signaling and tumor self-renewal ability with enhanced Dclk1 highlights the collective mechanism involved in tumor growth and survival. However, the precise mechanism by which Dclk1 supports intestinal tumor progression is poorly understood. With the aid of the *Apc* ^*Min/+*^ mouse model, we assessed the contribution of Dclk1 to intestinal tumorigenesis using small interfering RNAs targeting Dclk1 incorporated into poly(lactic-co-glycolic acid) nanoparticles (siDclk1-NPs). We found that Dclk1 is involved in enhancing the pro-survival signaling pathways and tumor cells’ self-renewal ability to facilitate intestinal tumor growth and progression.

RETRACTED

## Methods

### TCGA Colon Adenocarcinoma (COAD) Data

The RNA-seq datasets from February 2015 combining data from 329 patients with colon adenocarcinomas included in the Cancer Genome Atlas (TCGA) dataset were downloaded through the UCSC cancer genome browser (https://www.xenabrowser.net), as previously described [28].

### Determination of DCLK1-correlated pro-survival signaling in *APC* mutant COAD

*APC* mutant/*APC* non-mutant samples and samples with high/low DCLK1 expression levels were sorted by R v3.2. Patients whose DCLK1 expression levels was in the top 25% or bottom 25% were considered DCLK1-high or DCLK1-low, respectively. The corrplot function (R package corrplot) was used to confirm the correlation between the expression levels of DCLK1 and other genes. A heatmap was produced using the heatmap.2 function (R package gplots) [28].

### DCLK1 network with pro-survival signaling utilizing the GeneMANIA database

Datasets, including physical interactions, pathway, and genetic interactions, were collected from the public domain GeneMANIA database. The dataset relevant to DCLK1 and the pro-survival signaling network was produced from the GeneMANIA database (http://www.genemania.org).

### Animals

All animal experiments were performed with approval and authorization from the Institutional Review Board and the Institutional Animal Care and Use Committee at the University of Oklahoma Health Sciences Center (Oklahoma City, Oklahoma). *Apc* ^Min/+^ mice on the C57BL/6 J background were obtained from The Jackson Laboratory and were maintained by breeding *Apc* ^Min/+^ males to C57BL/6 J females. Mice were genotyped with a PCR assay to identify carriers of the *Min* allele of *Apc*. Same sex (male) C57BL/6 J *Apc* ^*Min/+*^ and *Apc* ^+/+^ littermates at 30 week of age were used in the present study. The average life span of *Apc* ^Min/+^ mice on the C57BL/6 J background is ∼ 20 weeks, although the mice in our facility have healthier survival, as observed in several previous studies [5–8]. *Apc* ^Min/+^ mice (i.e., >30 weeks of age) were carefully monitored and sacrificed before becoming moribund.

### Intestinal Epithelial Cell (IEC) Isolation

Small intestines (ileum) were attached to a paddle, were immersed in Ca^2+^-free standard Krebs-buffered saline (in mmol/l: 107 NaCl, 4.5 KCl, 0.2 NaH_2_PO_4_, 1.8 Na_2_HPO_4_, 10 glucose, and 10 EDTA) at 37 °C for 15–20 min, and were gassed with 5% CO_2_, 95% O_2_. Individual crypt units were then separated by intermittent (30 s) vibration into ice-cold phosphate buffered saline and were collected by centrifugation [18, 29–31]. We utilized the whole intestinal epithelilal cells.

RETRACTED

### FACS

Freshly isolated IECs were washed and resuspended in RPMI glutamax medium. To avoid endothelial and stromal contamination, isolated cells were incubated with anti-CD45, anti-CD31, anti-EpCAM, and anti-Dclk1 antibodies conjugated with the respective fluorochromes for 30 min. The cells were washed and sorted using an Influx-V cell sorter (Cytopeia). CD45^−^CD31^−^EpCAM^+^Dclk1^+^ cells were collected and then subjected to enterosphere formation assays [18, 30].

### Clonogenic assay

FACs isolated Dclk1^+^ IECs were plated in 48-well plates at a density of 100 cells per well in RPMI medium containing 0.3% soft agar. The cell suspensions were plated in a 48-well plate above a layer of solidified 1% soft agar in plain RPMI medium. The plates were incubated at 37 °C under 5% CO_2_. The cells were followed for enterosphere/enteroid formation, as described previously [18, 30, 31].

### RNA isolation and real-time RT-PCR analysis

Total RNA isolated from small intestinal epithelial cells was subjected to reverse transcription. The complementary DNA (cDNA) was subsequently used to perform real-time PCR with SYBR™ chemistry (Molecular Probes, Eugene, OR) using gene-specific primers for specific transcripts. The crossing threshold value assessed by real-time PCR was noted for the transcripts and normalized to β-actin.

### Immunoblot analysis

Twenty-five micrograms of the total protein was size-separated in a 4–12% SDS polyacrylamide gel and transferred electrophoretically onto a PVDF membrane with a wet-blot transfer apparatus (Bio-Rad, Hercules, CA). The membrane was blocked and incubated overnight with a primary antibody and was subsequently incubated with horseradish peroxidase-conjugated secondary antibody. The proteins were detected using ECL Western blotting detection reagents (Amersham-Pharmacia, Piscataway, NJ). Actin (42-kD) was used as a loading control.

### Small interfering RNAs

The Dclk1 siRNA (siDclk1; Cat. # S234357) sequence targeting the coding region of Dclk1 (accession No. NM_019978) and scrambled siRNAs (siScr; Cat. # AM4636) not matching any of the mouse genes were obtained (Ambion Inc., Austin, TX, USA). DCLK siRNA (h) (# SC45618), RELA siRNA (h) (#SC29410) and NOTCH1 siRNA (h) (#SC36095) were obtained from Santa Cruz Biotechnology (SCBT, TX, USA).

### Synthesis and characterization of Dclk1 siRNA NPs and treatment

Poly(lactide-*co*-glycolide acid nanoparticles (PLGA NPs) were synthesized using a double emulsion solvent evaporation technique, as described previously [18, 20]. The amount of encapsulated siRNA was quantified using a spectrophotometer (DU-800, Beckman Coulter, Brea, CA). The size, polydispersity index, and zeta-potential measurements of synthesized siRNA NPs were determined using diffraction light scattering (DLS) utilizing Zeta PALS (Brookhaven Instruments, Holtsville, NY). Sex- and age-matched littermates of C57BL/6 J *Apc* ^*Min/+*^ mice were injected i.p. with 0.25 nmol of siRNA preparation on every third day for a total of six doses.

RETRACTED

### Immunohistochemistry/immunofluorescence

Standard immunohistochemistry and immunofluorescence protocols were used with specific antibodies, as described previously [18, 30].

### Antibodies

We used the following antibodies: Dclk1, Lgr5, Bmi1, Hes1, Tcf4, Cox1, Cox2, EpCam, CD45, CD31 (all from Abcam, Cambridge, MA), CXCL1, CyclinD1, cMYC, β − catenin (Santa Cruz Biotechnology, USA), Notch1, NfkB-p65, CyclinD1, Ras, β-actin (Cell Signaling, Danvers, MA, USA), anti-rabbit IgG, anti-mouse IgG, anti-goat IgG (Jackson ImmunoResearch, West Grove, PA, USA), Alexa Fluor® 488 donkey anti-rabbit IgG, and Alexa Fluor® 568 donkey anti-goat IgG (Invitrogen, USA).

### siRNA-mediated knockdown of DCLK1

HT-29 and DLD1 human colon cancer cells were purchased from the American Type Culture Collection (ATCC) and were maintained in DMEM medium containing 10% fetal bovine serum (FBS). For siRNA-mediated knockdown studies, cells were seeded into 6-cm petri dishes and were allowed to attach overnight. After attachment, 25 nM of commercially validated siRNA targeting human DCLK1 or NOTCH1 or RELA (siRNA; Santa Cruz Biotechnology) or 25 nM human scrambled sequence (siSCR) not targeting any known genes were complexed with Lipofectamine 3000 (Invitrogen) and added to the dishes in fresh cell culture medium. After 48 h of treatment, cells were collected for migration, invasion, colony formation, and self-renewal (clonogenic) analysis.

### Migration and invasion assay

For the invasion assay, matrigel-coated Transwells (BD Biosciences) were prepared by retrieving in serum-free media for 2 h at 37 °C. For the migration assay, Transwells (BD Biosciences) were also used. Subsequently, HT-29 and DLD1 cells (5000/well) pre-transfected with either 25 nM siRNA or siSCR for 48 h were seeded into each Transwell in triplicate in serum-free media. Cell culture medium containing 10% FBS was added to the bottom of each well as chemoattractant, and the cells were incubated for 24 h at 37 °C under 5% CO_2_. Afterwards, a cotton swab was used to scrape non-invasive/migratory cells off the top of Transwells; the remaining cells were fixed with 100% methanol, stained with 0.1% crystal violet, and allowed to dry. After drying, all invading cells were counted from each Transwell. Results are reported as the number of cells invaded and/or migrated.

RETRACTED

### Colony formation assay

HT-29 and DLD1 were transiently transfected with si-DCLK1, siNFkB-p65, and si-NOTCH1 (from Santa Cruz Biotechnology), along with scramble siRNA. After 48 h, cells were seeded and passaged into new 6-well plates (100 cells/well). Cells were allowed to grow for one week, then were fixed with glacial acetic acid/methanol solution (1:3) and washed with PBS. Colonies were stained with 0.5% Crystal violet for 10 min and were washed with tap water to remove excess stain. Colonies were then counted under a stereomicroscope using a 1-cm^2^ grid. Four squares from four quadrants were counted for each well.

### Statistical analysis

Statistical analyses were conducted using GraphPad Prism 6.00 (GraphPad Software, La Jolla) and R system v3.2 for statistical computing. Pearson product–moment correlation was used for analysis and correlation of gene expressions between two groups. Colon cancer recurrence-free survival analysis was performed using Kaplan Meier Survival analyses. *P* values of <0.05 = *, <0.01 = **, and 0.001 = *** were considered statistically significant.

## Results

### DCLK1 is correlated with pro-survival signaling in colon adenocarcinoma

Mutation and/or loss of function of *APC* is the cause of more than 80% of colon cancers. DCLK1^+^ tumor stem cells are vital to the development and progression of colon cancer in *Apc* ^*Min/+*^ mice models. Indeed, the DCLK1 signature in *APC* mutant colon cancer predicts recurrence-free-survival (Additional file 1: Figure S1). Kaplan-Meier survival analysis demonstrated that the APC-derived DCLK1 signature could be used to strongly predict recurrence-free survival in colon cancer. The recurrence-free survival analysis of APC mutant patients with high DCLK1 expression (*n* = 31) tended to be associated with a poor prognosis compared with APC mutant patients with low DCLK1 expression (*n* = 35; *P* = 0.0171).

Although the DCLK1 expression levels are important in APC mutant colon cancer to predict the cancer stemness, the role of DCLK1 in regulating the prosurvival signaling pathways for intestinal cancer progression is largely unknown. Analysis of TCGA colon adenocarcinoma (COAD) cancer datasets demonstrated a strong correlation between DCLK1 mRNA expression and pro-survival signaling, including CTNNB1, NOTCH1, RELA, PTGS1, and PTGS2, as determined by the Pearson product–moment correlation, as previously described (Fig. 1a). DCLK1 was most strongly correlated with COX1 signaling in colon cancers (Additional file 2: Figure S2). Furthermore, heatmaps demonstrating dysregulated expression of the pro-survival signaling signature are higher in DLCK1-high patients than in DCLK-low patients from the TCGA COAD dataset (Fig. 1b). The GeneMANIA webserver was utilized to predict interactions between the DCLK1 and pro-survival signaling in the network using the parameters limited to physical interactions, genetic interactions, and pathways to score nodes and source organism *Homo sapiens* as additional parameters (Fig. 1c). From the GeneMANIA network, it is apparent that DCLK1 has networked with pro-survival signaling, and DCLK1 shows its interaction with pro-survival signaling via downstream factors/adaptor factors, exception is PTGS1 directly networking with DCLK1. These findings suggest that DCLK1 in colon cancers may have a relationship with pro-survival signaling and, by regulating pro-survival signaling, may assist in the development and progression of colon cancer.

RETRACTED

**Fig. 1:** DCLK1 expression is positively correlated with genes of pro-survival signaling pathways and tumor stem cell markers. **a** Color indicates correlation of DCLK1 and other genes: 1) negative (green), and 2) positive (red). **b** Heatmap of pro-survival signaling pathways and tumor stem cell markers gene expression levels by dividing colon cancer patients into two groups based on DCLK1 expression levels from TCGA. Patients with the top 25% or bottom 25% DCLK1 expression levels were considered DCLK1-high or DCLK1-low, respectively. **c** A gene network from GeneMANIA shows the relationships for genes from the list (nodes) connected (with edges) according to the functional association networks from the databases. Based on the physical interactions, pathway, and genetic interactions, in the network representation, all the nodes are connected and related to DCLK1

### *Apc*^*Min/+*^ mice with intestinal adenocarcinoma showed increased expression of tumor stem cells

Tumor stem cells (TSCs) are highly tumorigenic cells that have the ability to self-renew, giving rise to other malignant stem cells; TSCs are also phenotypically diverse cancer cells that are considered to be the source of tumor initiation and maintenance [32, 33]. To investigate the role of Dclk1^+^ TSCs in intestinal tumorigenesis under *Apc* mutation, we analyzed the level of Dclk1 expression and Dclk1^+^ cells in the intestines of *Apc* ^*Min/+*^ and wild-type (WT) mice. Compared with WT intestinal sections, the Dclk1 staining increased in *Apc* ^*Min/+*^ mouse intestines (Fig. 2a). The intensity of Dclk1 staining is 5–10 fold higher in the intestinal sections from *Apc* ^*Min/+*^ mice than those of WT mice (Fig. 2a and b). Furthermore, FACS analysis of the isolated IECs of *Apc* ^*Min/+*^ mice showed 25-30% Dclk1^+^ cells compared with 1-3% Dclk1^+^ cells from WT mice (Fig. 2c). We analyzed the expression of tumor stem cell markers, and found a massive increase in mRNA and protein levels of the Dclk1, Lgr5, Bmi1, and Musashi1 (Fig. 2d) in the IECs of *Apc* ^*Min/+*^ mice compared with WT control mice, corroborating the presence of highly tumorigenic cells in the Apc mutant intestinal tumors. Furthermore, FACS isolated Dclk1^+^ cells from *Apc* ^*Min/+*^ mice were utilized for Dclk1, Lgr5 and Bmi1 mRNA expression analysis and found that Dclk1^+^ cells are enriched with the tumor stem cell markers (Additional file 3: Figure S3).

RETRACTED

**Fig. 2:** Increased expression of Dclk1 and Dclk1^+^ cells in the intestinal adenomas and adenocarcinomas of *Apc* ^*Min/+*^ mice is associated with enhanced expression of tumor stem cell markers and pro-survival signaling. **a** IHC for Dclk1 in the small intestines of WT and *Apc* ^*Min/+*^ mice. **b** Staining intensity was scored and is represented as a bar graph. **c** FACS data representing the % Dclk1^+^ cells isolated from the small intestines of WT and *Apc* ^*Min/+*^ mice. **d** Differences in the number of Dclk1^+^ cells in staining and FACS corroborate with protein and mRNA levels of Dclk1 in the isolated IECs of WT and *Apc* ^*Min/+*^ mice; protein and mRNA levels analyzed by western blot and RT-PCR of Bmi1, Lgr5, and Musashi1 in isolated IECs from WT and *Apc* ^*Min/+*^ mice. **f** Protein expression levels of pro-survival signaling and their downstream targets in the isolated IECs of WT and *Apc* ^*Min/+*^ mice, analyzed by western blot. **e** mRNA expression levels of pro-survival signaling and their downstream targets in the isolated IECs of WT and *Apc* ^*Min/+*^ mice, analyzed by RT-PCR. All quantitative data are expressed as means ± *SD* of a minimum of three independent experiments. *P* values of <0.05 = *, <0.01 = **, and 0.001 = *** were considered statistically significant

### Amplified pro-survival signaling in the IECs of *Apc*^*Min/+*^ mice are critical for tumorigenesis

Pro-survival signaling pathways critical for cell survival and proliferation in IECs are required for adenoma and adenocarcinoma formation [34–36]. In contrast to normal intestinal epithelium, neoplastic cells have active pro-survival signaling pathways for proliferation, resistance, self-renewal, and survival [37, 38]. We detected greater expression of β-catenin, Notch, and phospho- and total NFκB-p65 in the IECs from *Apc* ^*Min/+*^ mice than in IECs from WT mice. The downstream targets COX1, COX2, CyclinD1, Tcf4, Ras, Hes-1, and CXCL1 were also upregulated in the IECs from *Apc* ^*Min/+*^ mice compared with IECs from WT mice (Fig. 2e and f). Thus, *Apc* loss may act as a primary window for the dysregulation of pro-survival signaling pathways to support the transformation of IECs towards neoplasia and promote progression. Further, these pro-survival signaling pathways are required for cell and stem cell homeostasis under non-neoplastic conditions; however, they can act as oncogenic factors for tumor maintenance and growth during neoplasia (24, 26).

RETRACTED

### Dclk1^+^ tumor stem cells from the intestines of *Apc*^*Min/+*^ mice are highly clonogenic, and the enteroids formed display increased pro-survival signals and stemness

FACS data revealed more Dclk1^+^ cells from the isolated IECs of *Apc* ^*Min/+*^ mice than from IECs of WT controls. Further, analysis of TCGA colon adenocarcinoma (COAD) cancer datasets demonstrated a correlation between DCLK1 mRNA expression and tumor stem cell markers LGR5 and BMI1, as determined by the Pearson product–moment correlation, as previously described (Fig. 1a). Furthermore, heatmaps demonstrating dysregulated expression of the tumor stem cell markers are higher in DLCK1-high patients than in DCLK-low patients from the TCGA COAD dataset (Fig. 1b).

From the GeneMANIA network, it is apparent that DCLK1 has networked with BMI1, and lacks a direct network with LGR5 within the limited parameters of interactions (Additional file 3: Figure S3). Therefore, we investigated whether Dclk1^+^ tumor stem cells with the *Apc* mutation have enriched co-expression of other tumor stem cell markers, and enhanced self-renewal, and pro-survival signaling pathways. Dclk1^+^ cells isolated from the small intestines of *Apc* ^*Min/+*^ mice formed a 5-fold increase in enteroids, which were also larger than the enteroids observed in WT mice (Fig. 3a and b). Next, we analyzed whether Dclk1^+^ enteroids of *Apc* ^*Min/+*^ mice are enriched with tumor stem cell markers and pro-survival signaling pathways. We collected Dclk1^+^ enteroids and analyzed them for the expression of tumor stem cell markers and pro-survival signaling pathways. We found enhanced Dclk1 expression in the enteroids of *Apc* ^*Min/+*^ mice compared with WT mice (Fig. 3c and d). Strikingly, the expression levels of Lgr5, Bmi1, and Musashi1 were significantly higher in the enteroids of *Apc* ^*Min/+*^ mice than in WT mice (Fig. 3c and d). These data suggest that this enhancement in Dclk1 expression, along with other tumor stem cell markers, may provide Dclk1^+^ cells with greater tumor stem cell function and self-renewal ability.

**Fig. 3:** Dclk1^+^ cells isolated from the IECs of *Apc* ^*Min/+*^ mice display enhanced self-renewal ability and enriched tumor stem cell markers and pro-survival signaling. **a** Enteroids formation of isolated Dclk1^+^ cells (100 cell per well) from the small intestines of WT and *Apc* ^*Min/+*^ mice. **b** Stacked bar and line graph represent the quantification of the number of enteroids formed and spheroid volume from the Dclk1^+^ cells isolated from WT and *Apc* ^*Min/+*^ mice. **c** & **d** mRNA and protein expression of Dclk1, Bmi1, Lgr5, and Msi1 in the isolated IECs of *Apc* ^*Min/+*^ mice compared with WT mice. **e** & **f** mRNA and protein expression of pro-survival signaling and their downstream targets in the isolated IECs of *Apc* ^*Min/+*^ mice compared with WT mice. All quantitative data are expressed as means ± *SD* of a minimum of three independent experiments. *P* values of <0.05 = *, <0.01 = **, and 0.001 = *** were considered statistically significant

We also collected the enteroids and examined the protein and gene expression of pro-survival signaling pathways. We found a significant increase in the expression of β-catenin, Notch1, and the NF-κB-p65 active form (phosphorylation at Ser536, Ser276) and total form in the enteroids of *Apc* ^*Min/+*^ mice compared with WT mice (Fig. 3e and f). Downstream targets cyclinD1, c-Myc, Tcf4, Ras, and Hes-1 were also increased in the enteroids of *Apc* ^*Min/+*^ mice compared with WT. Thus, the increased pro-survival signaling and tumor stem cell markers in the Dclk1^+^ enteroids may be the source for increased self-renewal ability and survival upon loss of *Apc* function.

RETRACTED

### Knocking down Dclk1 expression decreased the intestinal tumorigenesis in *Apc*^*Min/+*^ mice

Dclk1 expression levels and Dclk1-expressing cells are enhanced in the IECs of *Apc* ^*Min/+*^ mice. These findings suggest that Dclk1 may play a crucial role in development and progression of intestinal tumors under the loss of *Apc* function*.* To test our hypothesis that Dclk1 is required for intestinal tumorigenesis under the loss of *Apc* function, we inhibited *Dclk1* gene expression using siDclk1-NPs, along with si-Scramble-Nanoparticles (siScr-NPs) as a control, in *Apc* ^*Min/+*^ and WT mice. Histological observations of intestinal sections revealed fewer polyps and reduced dysplasia in the intestines of *Apc* ^*Min/+*^ mice treated with siDclk1-NPs compared with siScr-NPs (Additional file 4: Figure S4). Compared with siScr-NPs treatment, siDclk1-NPs treatment reduced the intensity of Dclk1 staining (~3fold) in intestinal sections from *Apc* ^*Min/+*^ mice (Fig. 4a). Furthermore, FACS analysis of Dclk1^+^ cells from the isolated IECs of *Apc* ^*Min/+*^ mice showed that siDclk1-NPs treatment significantly reduced the number of Dclk1^+^ cells compared with siScr-NPs treatment (Fig. 4b). Significantly lower expression of Dclk1 and the other tumor stem cell markers, Lgr5, Bmi1, and Musashi1, were detected in the isolated IECs of siDclk1-NP–treated *Apc* ^*Min/+*^ mice (Fig. 4c and d). However, expression of Bmi1 and Msi1 was either unchanged or increased in the siDclk1-NP–treated WT mice (Fig. 4c and d). No change in crypt architecture or abnormalities was observed in the WT mice treated with siDclk1-NPs or siScr-NPs as previously reported [18].

RETRACTED

**Fig. 4:** *Dclk1* knockdown reduced the expression of Dclk1 and Dclk1^+^ cells and the associated expression of tumor stem cell markers and pro-survival signaling in the *Apc* ^*Min/+*^ mice. **a** IHC for Dclk1 in the small intestines of *Apc* ^*Min/+*^ mice treated with siDclk1-NPs and siScramble-NPs; staining intensity was scored and represented as a bar graph. **b** FACS data representing the % Dclk1^+^ cells isolated from the small intestines of *Apc* ^*Min/+*^ mice treated with siDclk1-NPs compared with siScramble-NPs. **c** & **d** mRNA and protein expression levels of Dclk1, Bmi1, Lgr5, and Musashi1 in the isolated IECs of WT and *Apc* ^*Min/+*^ mice treated with siDclk1-NPs and siScramble-NPs, analyzed by RT-PCR and western blot. **f** Protein expression levels of pro-survival signaling and their downstream targets in the isolated IECs of WT and *Apc* ^*Min/+*^ mice, analyzed by western blot. **e** mRNA expression levels of pro-survival signaling and their downstream targets in the isolated IECs of WT and *Apc* ^*Min/+*^ mice, analyzed by RT-PCR. All quantitative data are expressed as means ± *SD* of a minimum of three independent experiments. *P* values of <0.05 = *, <0.01 = **, and 0.001 = *** were considered statistically significant

### Dclk1 regulates pro-survival signaling pathways to support intestinal tumorigenesis in *Apc*^*Min/+*^ mice

Conserved pro-survival signaling pathways, most notably the β-catenin, Notch, and NFkB pathways, coordinately regulate tumor formation and progression [34–36]. In the present study, we found that Dclk1^+^ cells isolated from the intestinal epithelium of *Apc* ^*Min/+*^ mice display enhanced expression of pro-survival signaling pathways and self-renewal ability (Fig. 3). To test whether Dclk1 regulates pro-survival signaling pathways in the isolated IECs from *Apc* ^*Min/+*^ mice, we silenced Dclk1 expression using siDclk1-NPs. Depleting Dclk1 in *Apc* ^*Min/+*^ mice had a potent inhibitory effect on the pro-survival β-catenin, Notch1, and NF-κB-p65 signaling pathways in the isolated IECs (Fig. 4e and f). To further clarify whether the inhibitory activity of β-catenin, Notch1, and NF-κB-p65 signaling caused by Dclk1 depletion is connected with an associated change in target gene expression, downstream targets COX1, COX2, CyclinD1, Tcf4, Ras, Hes-1, and Cxcl1 were quantified and were observed to be reduced in the IECs from *Apc* ^*Min/+*^ mice treated with si-Dclk1-NP (Fig. 4e and f).

RETRACTED

These data suggest that the Dclk1 expression level is indispensable for the activation of pro-survival signaling pathways upon loss of *Apc* function. However, the expression of pro-survival signaling was not altered in the IECs of WT mice treated with si-Dclk1-NP, except for a marginal increase in CyclinD1, suggesting that cell cycling may be controlled by Dclk1 expression levels (Fig. 4e and f). Together, knocking down Dclk1 decreased the pro-survival signaling in the IECs of *Apc* ^*Min/+*^ mice but not significantly in the WT mice.

### Dclk1 is required for intestinal tumorigenesis in *Apc*^*Min/+*^ mice

Stemness and self-renewal ability are the key features in tumorigenesis, for tumor initiation and progression [33]. To determine whether Dclk1 is critical for intestinal tumorigenesis, we inhibited *Dclk1* gene expression using siDclk1-NPs, along with siScr-NPs as control, in *Apc* ^*Min/+*^ mice. The self-renewal ability of Dclk1^+^ cells and their clonal populations is reduced with siDclk1-NP treatment, as evidenced by fewer and smaller enteroids formed from Dclk1^+^ cells of *Apc* ^*Min/+*^ mice (Fig. 5a-c). Next, we analyzed whether Dclk1^+^ enteroids of *Apc* ^*Min/+*^ mice treated with siDclk1-NP displayed diminished tumor stem cell markers and pro-survival signaling pathways. We found reduced Dclk1 expression in the enteroids of *Apc* ^*Min/+*^ mice treated with siDclk1-NP compared with siScr-NPs (Fig. 5d). Expression levels of Lgr5, Bmi1, and Musashi1 were also significantly reduced in the enteroids of *Apc* ^*Min/+*^ mice treated with siDclk1-NP (Fig. 5d).

**Fig. 5:** *Dclk1* knockdown in the *Apc* ^*min/+*^ mice reduced the stemness and pro-survival signaling of Dclk1^+^ cells. **a** Enteroids formation of isolated Dclk1^+^ cells (100 cell per well) from the small intestines of *Apc* ^*Min/+*^ mice treated with siDclk1-NPs and siScramble-NPs. **b** Stacked bar and **c** line graph represent the quantification of the number of enteroids formed and spheroid volume from the isolated Dclk1^+^ cells of *Apc* ^*Min/+*^ mice. **d** mRNA and protein expression of Dclk1, Bmi1, Lgr5, and Msi1 in the isolated IECs of *Apc* ^*Min/+*^ mice treated with siDclk1-NPs and siScramble-NPs. **e** & **f** mRNA and protein expression of pro-survival signaling and their downstream targets in the isolated IECs of *Apc* ^*Min/+*^ mice treated with siDclk1-NPs and siScramble-NPs. All quantitative data are expressed as means ± *SD* of a minimum of three independent experiments. *P* values of <0.05 = *, <0.01 = **, and 0.001 = *** were considered statistically significant

In addition, we examined the protein and gene expression of pro-survival signaling pathways and found that the expression of β-catenin, Notch1, and the NF-κB-p65 active form (phosphorylation at Ser536, Ser276) and total form in the enteroids of *Apc* ^*(Min/+)*^ mice treated with siDclk1-NP was less than the expression in mice treated with siScr-NP (Fig. 5e). Downstream targets cyclinD1, c-Myc, Tcf4, Ras, and Hes-1 were also reduced in the enteroids of *Apc* ^*(Min/+)*^ mice treated with siDclk1-NP (Fig. 5e). Together, these data suggest that Dclk1 is important and required for i) intestinal tumorigenesis, ii) increased stemness during neoplasia, and iii) increased pro-survival signaling to support tumor progression. Together, the present data suggests that Dclk1 knockdown downregulates pro-survival signaling, stemness, polyps, and, thus, tumorigenesis.

RETRACTED

### Silencing the pro-survival signaling Notch1 and RELA in human colon cancer cell lines reduced cancer cells’ self-renewal and progression

To further investigate whether DCLK1 regulates *APC* mutant colon tumorigenesis via pro-survival signaling pathways, we knocked down NOTCH1 and RELA in colon cancer cell lines and monitored for self-renewal and colony formation ability and migration and invasion in vitro. We utilized siRNAs against NOTCH1 and NF-κB-p65 (RELA) to deplete their gene expression in DLD1 and HT29 colon cancer cells. We also used siRNAs against DCLK1 in the colon cancer cells as a proportional strategy. Protein and mRNA expression analysis confirmed a significant decrease in NOTCH1, RELA, and DCLK1 protein and mRNA levels in cancer cells treated with the respective siRNAs (Fig. 6a). The effect of NOTCH1 and RELA knockdown on the self-renewal ability of DLD1 and HT29 cells was analyzed with a clonogenic assay. We found that the number of colonospheres formed was significantly reduced with siRNA treatment against NOTCH1 and RELA5 compared with the si-Scramble treatment (Fig. 6b). Indeed, DCLK1 knockdown showed higher inhibitory action on colon cancer cell self-renewal ability than NOTCH1 or RELA inhibition (Fig. 6b). Colon cancer cells’ colony-forming ability, which represents the cells’ viability and survival, was reduced in cells treated with siRNAs against NOTCH1 and RELA (Fig. 7a). Like colony formation, colon cancer cells’ in vitro migration and invasion were significantly reduced with siRNA treatment against Notch1 and NF-κB-p65, compared with si-Scramble treatment (Fig. 7b and c). However, the inhibitory effect of siNOTCH1 and siRELA on colon cancer cell colony formation and invasion/migration was less than the effect of siDCLK1 treatments (Fig. 7b and c). DCLK1 knockdown in colon cancer cells also reduced the mRNA expression levels of NOTCH1, RELA and ERK1/2 (Additional file 5: Figure S5). Finally to test the effect of MAPK inhibition in the regulation of BMI1 expression in the colon cancer cells, ERK1/2 siRNA was treated to the cells and found that their inhibition decreased the expression of BMI1 (Additional file 6: Figure S6). The present data suggest that pro-surivial signaling may support the colon cancer cell self-renewal and progression. Together, these results revealed that DCLK1 controls the pro-survival signaling pathways in colon cancer cells to support the survival and stemness of tumor cells vital for their progression.

RETRACTED

**Fig. 6:** Silencing *DCLK1* and pro-survival signaling NOTCH1 and RELA reduce the self-renewal ability of human colon cancer cells (DLD1 & HT29). **a** Protein and mRNA expression levels of DCLK1, NOTCH1, and RELA in the DLD1 and HT29 colon cancer cells transfected with si-DCLK1, si-NOTCH1, and siRELA compared with siScramble-transfected cells. **b** Self-renewal ability of DLD1 and HT29 cells after the knockdown of DCLK1, NOTCH1, and RELA; bar graph represents the average number of spheroids formed from DLD1 and HT29 cells after the knockdown of DCLK1, NOTCH1, and RELA. All quantitative data are expressed as means ± *SD* of a minimum of three independent experiments. *P* values of <0.05 were considered statistically significant

**Fig. 7:** Silencing *DCLK1* and pro-survival signaling reduced the survival ability of human DLD1 & HT29 colon cancer cells. **a** Colony formation ability of DLD1 and HT29 cells after the knockdown of DCLK1, NOTCH1, and RELA; bar graph represents the average number of colonies formed from DLD1 and HT29 cells after the knockdown of DCLK1, NOTCH1, and RELA. **b** In vitro invasion and migration of DLD1 cells after the knockdown of DCLK1, NOTCH1, and RELA; bar graph represents the number of cells migrated and invaded after the knockdown of DCLK1, NOTCH1, and RELA. **c** In vitro invasion and migration of HT29 cells after the knockdown of DCLK1, NOTCH1, and RELA, bar graph represents the number of cells migrated and invaded after the knockdown of DCLK1, NOTCH1, and RELA. All quantitative data are expressed as means ± *SD* of a minimum of three independent experiments. *P* values of <0.05 were considered statistically significant

## Discussion

Our previous studies demonstrated that Dclk1 overexpression is correlated with intestinal cancer progression and that silencing Dclk1 decreased the number and size of polyps, adenoma, and adenocarcinoma, suggesting that Dclk1 plays an important active role in intestinal tumorigenesis [18, 28, 39, 40]. Tumor cell self-renewal and survival ability are the key features in tumorigenesis, for tumor progression [33]. Pro-survival signaling pathways, most notably the ß-catenin, Notch, and NFkB pathways, coordinately regulate tumor cell survival and self-renewal [34–36]. However, whether Dclk1 regulates intestinal tumor cell survival and self-renewal for tumorigenesis through pro-survival signaling pathways is largely unknown. In the present study, we used *Apc* ^*Min/+*^ mice, an excellent model to evaluate human FAP and sporadic colorectal cancer [1, 2, 7]. Consistent with our previous studies, we found increased expression of Dclk1 in the IECs of *Apc* ^*Min/+*^ mice, which exhibit high-grade dysplasia and adenocarcinoma [12, 18, 20]. It has been suggested that stem-like cells or stem cells are more abundant in cancerous conditions, and that the loss of *Apc* function increases the expansion of the tumor stem cell (TSC) compartment [3, 41]. Loss of *Apc* function significantly increased the expression of tumor stem cell markers Dclk1, Lgr5, Bmi1, and Musashi in the IECs. However, how loss of *Apc* selects the cell type or stem cell type in the process of tumorigenesis is yet to be identified. *Apc* regulates the *Wnt* signaling, which is critical for the maintenance of Lgr5+ stem cells and initiation and progression of cancer [3]. It is recently reported that Lgr5^+^ stem cells give rise to Dclk1^+^ cells in the intestinal epithelium [13]. Therefore, we suggest that the loss of *Apc* may induce the specific expansion of Lgr5^+^ cells derived Dclk1^+^ cells for intestinal tumorigenesis. However, the expansion of other stem cells and the specific expansion of Dclk1^+^ cells need to be investigated in future. We also observed enhanced self-renewal ability of Dclk1^+^ cells isolated from the intestines of *Apc* ^*Min/+*^ mice.

RETRACTED

Cellular pro-survival signaling pathways are interconnected, complex signaling networks, and their upregulation is well illustrated in cancers [42]. The aberrant upregulation or constitutive activation of multiple survival-signaling pathways in cancer cells promotes proliferation and stemness, inhibits apoptosis, and increases survival and the ability to invade and migrate into surrounding tissues and metastasize to distant sites [42, 43]. We found here that the ß-catenin, Notch, and NFkB pro-survival signaling pathways are upregulated in the isolated IECs of *Apc* ^*Min/+*^ mice. We further determined that Dclk1^+^ cells of *Apc* ^*Min/+*^ mice display enhanced pro-survival signaling pathways, compared with Dclk1^−^ cells. These findings suggest that the enhanced pro-survival signaling pathways could be a vital factor for tumor progression by regulating tumor stem cells and/or tumor cell stemness. Several studies have indicated that Dclk1 promotes the multistep process of cancer formation and progression [13, 18, 31, 40, 44–46]. It has been suggested that Dclk1 can regulate pluripotency factors, miRNAs, and signaling pathways, including NOTCH and Runx2, in cancer and non-cancer cells [46–48]. In the present study, we witnessed a similar phenomenon; the pro-survival signaling pathways were upregulated in the IECs of *Apc* ^*Min/+*^ mice, in which Dclk1 expression is higher than in controls. We observed that silencing Dclk1 reduced the pro-survival signaling pathways in the IECs of *Apc* ^*Min/+*^ mice. We have previously demonstrated that downregulation of DCLK1 can up-regulate critical miRNAs in both in vitro and in vivo cancer models and resulted in decreased pro-survival signaling and EMT-related transcription factors [13, 20, 44, 47]. Indeed, the enterospheres formed from the isolated Dclk1^+^ cells of *Apc* ^*Min/+*^ mice treated with si-Dclk1-NPs display reduced pro-survival signaling pathways, which may be the reason for reduced self-renewal and tumor stem cells.

We further investigated the connection between pro-survival signaling pathways and Dclk1 expression in the *Apc* ^*Min/+*^ mice with high-grade dysplasia and intramucosal adenocarcinoma. We observed that inhibition of NOTCH and RELA reduced the colon cancer cell lines DLD1 and HT29 self-renewal ability, survival/viability, and invasion/migration in vitro. However, DCLK1 knockdown is highly effective at inhibiting the self-renewal, colony formation, and invasion/migration of colon cancer cells than the NOTCH or RELA inhibition in vitro. Furthermore, DCLK1 knockdown decreased the expression of NOTCH, RELA and MAPK in colon cancer cells, suggesting that DCLK1 may act as a master regulator for multiple pro-survival signaling pathways, which could explain why any individual knockdown of pro-survival signaling is less effective than DCLK1 knockdown in inhibiting cancer cells’ self-renewal and progression. Our findings suggest that Dclk1 can regulate multiple signaling pathways for cancer formation and progression. However, the exact regulation mechanism of Dclk1 requires further clarification.

## Conclusions

In conclusion, we found that Dclk1 was enhanced in *Apc* mutant intestinal tumors, and elevated tumor stemness and survival by regulating the pro-survival signaling pathways. We also determined that Dclk1 knockdown reduced tumor stemness, polyps, adenoma, and adenocarcinoma by inhibiting pro-survival signaling and suppressing their downstream oncogenes. Together, these results suggest that Dclk1, a tumor stem cell marker, may be a potential therapeutic target for colon cancer therapy.

RETRACTED

## Additional files

Additional file 1: Figure S1. DCLK1 gene expression predicts survival in APC mutant colon cancer. (TIF 9612 kb)
Additional file 2: Figure S2. DCLK1 expression was positively correlated to COX1 signaling. (TIF 7698 kb)
Additional file 3: Figure S3. (**a**) Gene enrichment analysis in the FACs isolated Dclk1+ and Dclk1- of Apc^*Min/+*^ mice small intestine. (**b**) Network of Dclk1 with BMI derived from GeneMANIA. (TIF 7440 kb)
Additional file 4: Figure S4. DCLK1 knockdown decreased the intestinal tumorigenesis. (TIF 6996 kb)
Additional file 5: Figure S5. DCLK1 knockdown decreased the mRNA levels of NOTCH1, RELA and ERK1/2 in colon cancer cell lines. (TIF 6101 kb)
Additional file 6: Figure S6. ERK1/2 knockdown decreased the mRNA levels of BMI1 in DLD1 colon cancer cell line. (TIF 7467 kb)

## Abbreviations

Apc: *Adenomatous polyposis coli*
ATCC: American type culture collection
cDNA: Complementary DNA
COAD: Colon adenocarcinoma
CRC: Colorectal cancer
CSCs: Cancer stem cells
Dclk1: Doublecortin-like kinase1
EMT: Epithelial mesenchymal transition
FAP: Familial adenomatous polyposis
IECs: Intestinal epithelial cells
IHC: Immunohisto chemistry
PLGA: Poly(lactide-co-glycolide acid)
siDclk1-NPs: Si-Dclk1-Nanopartilces
siRNA: Small interference RNA
siScr-NPs: Si-Scramble-Nanoparticles
TCGA: The cancer genome atlas
TSCs: Tumor stem cells
